The article "Application of Internet of Things and Naive Bayes in Public Health Environmental Management of Government Institutions in China" was retracted in 2023. Reasons: unreliable results or conclusions; concerns about the data; concerns about the peer review; concerns about the citations.

# Application of Internet of Things and Naive Bayes in Public Health Environmental Management of Government Institutions in China

**DOI:** 10.1155/2021/9171756

**Published:** 2021-08-13

**Authors:** Zhipeng Zhang, Shuxiang Zhang

**Affiliations:** School of Politics and Public Administration, Zhengzhou University, Zhengzhou 450001, China

## Abstract

As the builder and maintainer of the city appearance and environment, the city appearance and environmental service industry provides urban residents with a beautiful, livable, and comfortable living environment and is also responsible for providing city appearance and environmental public health services for the economic and social functions carried by the global cities task. Based on this problem, this study has carried out the work of government agencies' public health environmental management and influencing factors based on the Internet of Things and edge computing. This study analyzes the influencing factors of public health environmental management of government agencies based on traditional research and conducts data analysis through the Naive Bayes algorithm. On this basis, the study combines the Internet of Things technology to construct system architecture for public health environmental management. The proposed management system is used to manage government agencies, which meets security, privacy and efficiency, and data security requirements. Experimental results prove that after algorithm optimization and architecture design, the evaluation level of the public health environment is significantly improved.

## 1. Introduction

The faster the pace of urbanization, the more problems will arise in the management of urban public environmental sanitation. Instead of using orthodox methods, problems in a new era with a new background need to be analyzed and solved using novel methods. Public environmental sanitation is one of the key tasks of urban governance [1, 2]. The task is to accelerate the transformation of service methods and better serve the economic construction of new areas. It assists urban governance in developing better and faster in the rapid development of cities that requires deeper discussions. Today's society has entered the information age [3]. Whether the public health and environmental management work of government agencies can keep up with the requirements of the times and whether it can meet the requirements of informatization has put forward requirements for the management of public social management [4].

It is vital to increase public health environmental management of government agencies in response to public demand [5]. With the expansion of the jurisdiction of the public health environment and the continuous health needs of residents and in order to maximize the utilization of health management resources, the improvement of health management is on the agenda. In order to integrate information resources and public social resources, it is feasible to use an integrated information management platform, which makes it possible to realize the unified management of public health [6, 7]. Zander assessed the degree of collaboration among multiple public health service providers in Wisconsin [8]. The coordination of multiple public health service supply organizations is widely used in the provision of various public health services, including tobacco prevention and control, maternal and child health, emergency planning, community assessment and planning, and immunization, according to the authors [9–11]. However, the environmental sanitation industry lacks systematic and theoretical research results. With the acceleration of our country's urbanization process, the contradiction between the public environment of government agencies and the people's growing expectations of life has become increasingly prominent. It has become a severe problem that plagues local governments. How may the management of this industry be improved? In comparison to other public utilities and public services, the use of systematic research and theory to assist and guide the sector is more practical [12, 13].

The article "Application of Internet of Things and Naive Bayes in Public Health Environmental Management of Government Institutions in China" was retracted in 2023. Reasons: unreliable results or conclusions; concerns about the data; concerns about the peer review; concerns about the citations.

With the development of network technology, merging social and public utilities with network technology has become possible. The use of computer information technology and using modern information management systems, on the one hand, can reduce the number of managers and save management time [14–16]. On the other hand, to a certain extent, it can save the labor cost of public social utilities, improve the staff's work efficiency, and improve the economic benefits of society. This article has carried out the work of government agencies' public health environmental management and influencing factors based on the Internet of Things and edge computing and utilizing Naïve Bayes algorithm for further data analysis in response to this challenge. The technology is based on health management indicators. It uses analytical methods to give detailed, accurate, and scientific information for public health environmental management decision-making. It also can track and evaluate anomalous signs.

The rest of the study is organized as follows. First, in Section 2, related technologies are discussed in detail. Then, in Section 3, the proposed scheme and the applications of Naive Bayes in healthcare management are studied, followed by government agency public health environmental management model in Section 4. Finally, the study is concluded in Section 5.

The article "Application of Internet of Things and Naive Bayes in Public Health Environmental Management of Government Institutions in China" was retracted in 2023. Reasons: unreliable results or conclusions; concerns about the data; concerns about the peer review; concerns about the citations.

## 2. Related Technologies

We are here to elaborate on the related developments of public health environmental management of government agencies, such as Internet of Things technology, to facilitate the follow-up research.

### 2.1. Research on Internet of Things Technology

The Internet of Things covers many fields, involves a wide range of networks, and the research content is complex and diverse [17]. Now, we analyze the typical application scenarios, discuss whether the existing solutions achieve security, privacy, and efficiency, and make some corresponding solutions. The Internet of Things is based on the existing Internet architecture. It expands it, so that the physical world can be interconnected with the virtual world [18, 19].  Figure 1 shows one of the typical architectures of Internet of Things technology.

With the construction of the Internet of Things infrastructure and the adjustment of web standards, more and more physical devices are connected to the Internet. As a result, the number of Internet of Things services is increasing [20–22]. Therefore, finding the required service objects from the vast number of Internet of Things services has gradually become a significant challenge for the Internet of Things applications. Furthermore, considering government agencies' data privacy and security, the Internet of Things technology can assist in public environmental management.

### 2.2. Public Health Environmental Management of Government Agencies

There are different modes of supply of public services. Public service providers can be government departments, nonprofit organizations, private individuals, market organizations, and international organizations [23, 24]. The supply model includes the cooperative supply model of the public and private sectors (public-private partnership model of public product supply), the complementary model of the government and the third party, the ternary subject cooperation model (the government, the market, and the voluntary sector jointly supply), and the cooperative supply of multiple subjects. Public environmental sanitation is one of the critical tasks of urban governance. How to accelerate the transformation of service methods, better serve the economic construction of new districts, and assist urban governance in developing better and faster in cities' rapid development need a more profound discussion [25]. It is necessary to seize opportunities further, change methods, innovate management methods, and adapt to new problems and new contradictions in the new situation.

## 3. Application of Naive Bayes in the Management of Public Health Environment in Government Agencies

In the discussion in the previous section, we believe that a set of information management systems suitable for public health environmental management of government agencies is necessary. It can manage public environmental big data, give critical information to public health management decision-makers, and provide information assistance. In the data processing stage, we use the Naive Bayes algorithm to analyze the data collected by the IoT system [26].

The article "Application of Internet of Things and Naive Bayes in Public Health Environmental Management of Government Institutions in China" was retracted in 2023. Reasons: unreliable results or conclusions; concerns about the data; concerns about the peer review; concerns about the citations.

The Naive Bayes classifier is based on the assumption of conditional independence and is widely used in actual production [27–29]. Substituting the independent assumption of attribute conditions, the Naive Bayes classifier integrates the relevant information provided by the data, prior knowledge, and unobserved variables and has higher accuracy.

(1) $$\begin{array}{c} E\left(v,h;\theta \right)=-\sum_{ij}W_{IJ}v_{i}h_{j}-\sum_{i}b_{i}v_{i}-\sum_{j}a_{j}h_{j}. \end{array}$$

It is not feasible to estimate a complete posterior probability, so this section introduces a variation method to approximate the posterior distribution.

(2) $$\begin{array}{c} P_{\theta }\left(v,h\right)=\frac{1}{Ζ\left(\theta \right)}\exp\left(-E\left(v,h;\theta \right)\right), \end{array}$$

where Ζ(*θ*) is the normalization factor called partition function.

The main idea is to construct a simple mathematical form for a particular model to approximate the posterior distribution of unobserved variables and give the lower bound of the marginal likelihood of the observed data [30–32]. Then, the integration process can be turned into a problem of finding the optimal value of the lower bound.

(3) $$\begin{array}{c} P_{\theta }\left(v,h\right)=\frac{1}{Ζ\left(\theta \right)}\exp\left(\sum_{i=1}^{D}\sum_{J=1}^{F}W_{ij}v_{i}h_{j}+\sum_{i=1}^{D}v_{i}b_{i}+\sum_{j=1}^{F}a_{j}h_{j}\right). \end{array}$$

The posterior probability is a more realistic probability obtained by combining the investigation evidence to obtain new additional information and correcting the prior probability [33]. The posterior probability reflects the ability of people to learn from observations. The posterior probability is also exhaustive.

(4) $$\begin{array}{c} P_{\theta }\left(v\right)=\frac{1}{Ζ\left(\theta \right)}\underset{h}{\sum }\exp\left[v^{T}Wh+a^{T}h+b^{T}v\right],\\ L\left(\theta \right)=\frac{1}{N}\overset{N}{\underset{\text{n}=1}{\sum }}\log\;P_{\theta }\left(v^{\left(n\right)}\right). \end{array}$$

In classification problems, there are usually objectives to be considered for classification, and appropriate decision-making criteria can be selected according to the purpose of classification. Commonly used decision-making rules include the minimum error rate criterion and the minimum risk criterion [34].  Figure 2 shows a schematic diagram of the data flow of the Naive Bayes algorithm.

(5) $$\begin{array}{c} \left(P,v|h\right)=\prod_{i}P,v_{i}|h\left(\right)P,v_{i}=1|h\left(\right)\\ =\frac{1}{1+\exp\left(-\sum_{j}W_{ij}h_{j}-b_{i}\right)},\\ \frac{\text{d}x^{\left(1\right)}}{\text{d}t}+ax^{\left(1\right)}=b,\\ \frac{\text{d}x}{\text{d}t}=\underset{\Delta t⟶0}{\lim}\frac{x\left(t+\Delta t\right)-x\left(t\right)}{\Delta t}. \end{array}$$

In classification problems, people often want to minimize classification errors. Starting from this requirement, the lowest error rate can be obtained [35]. Therefore, it is the minimum error rate criterion, which can be expressed as follows.

(6) $$\begin{array}{c} \frac{\Delta x}{\Delta t}=\frac{x\left(k+1\right)-x\left(k\right)}{k+1-k}\\ =x\left(k+1\right)-x\left(k\right)\\ =a^{\left(1\right)}\left[x\left(k+1\right)\right],\\ cv\left(b_{0}\right)=\underset{b>0}{\min}cv\left(b\right). \end{array}$$

The assumption of Bayesian decision-making is under the condition that the prior probability and conditional probability are known. However, under normal circumstances, the prior probability and conditional probability distribution are both unknown. Therefore, it needs to be based on the prior probability and the prior probability of the known sample pair. Therefore, the conditional probability distribution is estimated as

(7) $$\begin{array}{c} \Psi_{x}\left(\omega \right)=\ln\;\Phi_{x}\left(\omega \right)\\ =-\frac{1}{2}\omega^{2}\sigma^{2},\\ cv\left(b\right)={\sum_{i=1}^{n}\left[y_{i}-\overset{\wedge }{y_{\neq i}\left(b\right)}\right]}^{2}. \end{array}$$

Although the Bayesian network allows specific dependencies between class attributes, it also needs to make an initial assumption about the network structure, which also assumes a certain degree of conditional independence [36]. In addition, the reasoning process of the Bayesian network is very time-consuming. Cooper proved that using unconstrained Bayesian networks for probabilistic reasoning is an NP-hard problem [3].

The article "Application of Internet of Things and Naive Bayes in Public Health Environmental Management of Government Institutions in China" was retracted in 2023. Reasons: unreliable results or conclusions; concerns about the data; concerns about the peer review; concerns about the citations.

## 4. Government Agency Public Health Environmental Management Model Test

### 4.1. IoT Architecture Test Plan

In order to verify the superiority of the scheme in this study, this chapter tests the experiment of the scheme based on Java language. In the process, the commons-codec package based on Java language is used for coding calculation. The generation of base and exponent mainly depends on the KeyPairGenerator tool [37, 38]. This experiment mainly focuses on testing the four standard exponential lengths of 128 bit, 256 bit, 512 bit, and 1024 bit. Considering that the base length generally does not exceed the exponential length, the base lengths involved in the experiment are also 128 bit, 256 bit, 512 bit, and 1024 bit, which increase successively, and the value is random. In order to avoid errors caused by too few experiments, the experiment also uses multiple sampling to calculate the average value.

### 4.2. Effect Analysis of the Environmental Management Model

Environmental public service is a basic management function provided by the government as a social manager. The application of data by government departments reflects the government's decision-making level. The key to the feasibility of a big data intervention evaluation system is to be able to use big data technology to quantify the evaluation factors and complete the visual analysis of the factors.  Figure 3 shows the results of differential data for the public health environment.  Figure 4 describes the distribution results of environmental differences in government agencies.

This study uses big data to quantify some vitality evaluation factors. However, for vitality factors that cannot be quantified with big data, only traditional data can be used to quantify the suitability of the environment and the participation of landscape sketches. Therefore, in the future research process, it is necessary to dig in-depth data. Therefore, it is recommended that governments and departments at all levels reasonably disclose part of the data following the law. Also, the use of big data is to quantify more vitality factors, so that the vitality evaluation system is more accurate, rational, and reasonable.

From the differential data results of the public health environment shown in Figure 3, we can see that the Internet of Things architecture established in this article can effectively count and analyze the health environment. The results of the distribution of environmental differences in government agencies described in Figure 4 show the environmental differences between different government agencies. Obtaining high-accuracy environmental information data is a prerequisite for practical analysis.

In the process of applying and analyzing environmental systems, the critical step is to collect environmental data information. The city appearance and environmental service industry, as the builder and maintainer of city appearance and environment, provides urban residents with a beautiful, livable, and comfortable living environment and provides city appearance. In addition, the environmental public health services for the economic and social functions are carried out by global cities. To obtain accurate and comprehensive environmental data information, it is necessary to make full preparations. These include installing video monitors and specific placement points for sensors, selecting the monitoring range of the observation point, and checking whether the environmental information of the monitoring point is in a natural state and is not created deliberately. Only by eliminating unnecessary interference factors, we can obtain accurate and reliable information when collecting data and information, which is also a prerequisite for effective public governance of the environment. The classification of public environment types of government agencies is shown in Figure 5. The distribution of monthly visitors to the public health environment is shown in Figure 6.

The article "Application of Internet of Things and Naive Bayes in Public Health Environmental Management of Government Institutions in China" was retracted in 2023. Reasons: unreliable results or conclusions; concerns about the data; concerns about the peer review; concerns about the citations.

From the classification of the public environment types and the number of visitors shown in Figures 5 and 6, we consider the aggregation and changes of the flow of people from the perspective of the Internet of Things data to avoid considering only a single node. We can quickly establish where the most people collected in the entire area and where the fewest people gathered by analyzing big data. Numerical values can be used to quantify the degree of change and aggregation properly. Traditional data can only be based on the number of persons passing through a given node, where a fair amount of ambiguity may exist. With the free and widespread use of mobile phone signals in big data, we will be able to understand individuals in the future fully. The rule of behavior and stay time in public areas and the position and timing of crests and troughs where people congregate will all aid in the design of public spaces. Environmental public service is a basic management function provided by the government as a social manager. With the rapid development of society and the acceleration of urbanization, the public environment is becoming increasingly fragile, the ecosystem is constantly degrading, and environmental pollution is becoming more serious. Environmental problems have gradually become an important topic related to people's livelihood, especially in the scope of our activities. Appropriate and effective governance is more important for cities that have more impact on the public environment. The application of data by government departments reflects the government's decision-making level.

## 5. Conclusion

Public health environmental management of government agencies is the top priority in a public environment, and informatization construction puts forward requirements on relevant agencies. With the development of socialization of public health environmental management, the public health management model of informatization and information disclosure has become the management model pursued by modern institutions. As the builder and maintainer of the city's appearance and environment, the city's appearance and environmental service industry provide urban residents with a beautiful, livable, and comfortable living environment. It also shoulders the task of providing city appearance and environmental public health services for global cities' economic and social functions. Based on the Internet of Things and edge computing, this study has carried out the work of government agencies' public health environmental management and influencing variables. According to experimental data, the evaluation level of the public health environment has been greatly enhanced as a result of algorithm optimization and architecture design. However, due to the rapid development of the Internet of Things architecture system, the system's functions have not been able to cover all the public health management of government agencies. The improvement of the system's functions should be the focus of future maintenance. In addition, we will continue to devote ourselves to the research and further exploration of public health environmental management to provide a scientific reference for the management work of related institutions.

The article "Application of Internet of Things and Naive Bayes in Public Health Environmental Management of Government Institutions in China" was retracted in 2023. Reasons: unreliable results or conclusions; concerns about the data; concerns about the peer review; concerns about the citations.

## Figures and Tables

**Figure 1:** Typical architecture of IoT technology.

**Figure 2:** Schematic diagram of the data flow of the Naive Bayes algorithm.

**Figure 3:** Differential data results of public health environment.

**Figure 4:** Distribution of environmental differences in government agencies.

**Figure 5:** Classification of public environment types of government agencies.

**Figure 6:** Distribution of monthly visitors to the public health environment.

## Data Availability

The data used to support the research results of this study are available in public channels.
